RETRACTED

# GATA4 Regulates Inflammation-Driven Pancreatic Ductal Adenocarcinoma Progression

**DOI:** 10.3389/fcell.2021.640391

**Published:** 2021-04-29

**Authors:** Weiliang Jiang, Congying Chen, Li Huang, Jie Shen, Lijuan Yang

**Affiliations:** ^1^Department of Gastroenterology, Shanghai General Hospital, Shanghai Jiao Tong University School of Medicine, Shanghai, China; ^2^Shanghai Key Laboratory of Pancreatic Disease, Institute of Pancreatic Disease, Shanghai Jiao Tong University School of Medicine, Shanghai, China

**Keywords:** GATA4, pancreatic ductal adenocarcinoma, inflammation, LPS, tumor-associated macrophage

## Abstract

Cancer-associated inflammation is a key molecular feature in the progression of pancreatic ductal adenocarcinoma (PDAC). GATA4 is a transcription factor that participates in the regulation and normal development of several endoderm- and mesoderm-derived tissues such as the pancreas. However, it remains unclear whether GATA4 is involved in the inflammation-driven development of pancreatic cancer. Here, we employed quantitative reverse transcription PCR, immunohistochemistry, and differential expression analysis to investigate the association between GATA4 and inflammation-driven PDAC. We found that overexpression of GATA4 in pancreatic tumor tissue was accompanied by increased levels of inflammatory macrophages. We used macrophage-conditioned medium to validate inflammation models following treatment with varying concentrations of lipopolysaccharide and determined whether GATA4-dependent inflammatory stimuli affected pancreatic cancer cell invasion and growth *in vitro*. Nude mouse models of dibutyltin dichloride-induced chronic pancreatitis with orthotopic tumor xenografts were used to evaluate the effect of the inflammatory microenvironment on GATA4 expression *in vivo*. Our findings indicate that overexpression of GATA4 dramatically aggravated inflammatory stimuli-induced pancreatic cancer cell invasion and growth via NF-κB and STAT3 signaling, whereas silencing of GATA4 attenuated invasion and growth. Overall, our findings suggest that inflammation-driven cancer progression is dependent on GATA4 expression and is mediated through the STAT3 and NF-κB signaling pathways.

## Introduction

Pancreatic ductal adenocarcinoma (PDAC) is reportedly the twelfth most frequently occurring cancer in the world with the seventh highest mortality rate (Simoes et al., 2017). The high mortality rate is due to late presentation of symptoms as well as a high rate of reoccurrence in those patients that receive surgical resection (Tesfaye and Philip, 2019). The exact etiology of PDAC is not well understood but inflammation and pancreatitis are thought to be contributing factors (Lowenfels et al., 1993; Gukovsky et al., 2013; Lin and Zhang, 2017; Kong et al., 2018).

RETRACTED

Although the development of PDAC is associated with mutations in several pathways (Saiki and Horii, 2014), oncogenic KRAS mutations have been found in 90% of patients with PDAC and are considered to be essential to pancreatic carcinogenesis (Jones et al., 2008). However, since KRAS mutations also appear in populations without pancreatic cancer, carcinogenesis is likely to involve other factors besides KRAS mutations. One such factor is the inflammatory microenvironment (Sharma and Kanneganti, 2016). A study in mice discovered that the combination of an inflammatory microenvironment and oncogenic KRAS were found to induce carcinogenesis (Guerra et al., 2007). When challenged with pancreatitis, adult mice that had become resistant to KRAS^*G*12V^-induced PDAC developed the full invasive form of the disease. In addition, it is clear that inflammation accelerates the onset of PDAC in the presence of oncogenic Kras (Carrière et al., 2009). Furthermore, the transition from pancreatitis to cancer is promoted by the actions of proinflammatory mediators directly on cells that harbor KRAS mutations (Guerra et al., 2011; Loncle et al., 2015; Siddiqui et al., 2018). Specifically, the cytokine IL-6 induces expression and activation of signal transducer and activator of transcription 3 (STAT3), which is also upregulated by oncogenic KRAS (Steele et al., 2016; Wörmann et al., 2016; Van Gorp and Lamkanfi, 2019). Constitutive STAT3 signaling is associated with several cancers and plays an essential role in KRAS-induced pancreatic tumorigenesis (Corcoran et al., 2011). Moreover, JAK–STAT3 pathway activation correlates with a poor outcome in PDAC patients following resection (Denley et al., 2013). The PI3K pathway has also been shown to promote PDAC induced by oncogenic Kras through the activation of STAT3 and NF-Kb (Baer et al., 2014). Thus, inflammation that drives activation of multiple signaling pathways can promote the development of PDAC.

GATA4 is a member of the GATA zinc-finger transcription factor family. GATA binding motifs are found in a large number of gene promoters. GATA4 is involved in the normal development of several endoderm- and mesoderm-derived tissues, including the pancreas (Carrasco et al., 2012; Xuan and Sussel, 2016). GATA4 is expressed in the developing endocrine pancreas and activates glucagon gene expression (Ritz-Laser et al., 2005). Deletion of GATA4 in combination with GATA6 results in severe disruption of pancreatic progenitor cell proliferation in mice whereas single deletions of both genes have a relatively mild impact (Carrasco et al., 2012; Xuan et al., 2012), suggesting that both GATA6 and GATA4 are required during pancreatic development. More recently, GATA6 and GATA4 have been implicated in the regulation of foregut endodermal fates through the inhibition of GATA4/6-mediated hedgehog signaling (Xuan and Sussel, 2016).

RETRACTED

Although GATA4 is overexpressed in PDAC (Karafin et al., 2009), and GATA6-dependent dedifferentiation of acinar cells is known to influence KRAS-induced pancreatic cancer progressio (Hermann et al., 2014), the role of GATA4 during inflammation-related PDAC progression remains unclear. In this study, we observed high GATA4 expression levels in pancreatic tumor tissues together with an increased presence of inflammatory macrophages. We established an inflammatory model *in vitro* using macrophage-conditioned medium (MCM) and varying concentrations of lipopolysaccharide (LPS), and assessed whether GATA4 was involved in inflammatory stimuli-induced pancreatic cancer cell invasion and growth. We also examined whether GATA4 expression influences cancer progression through associations with inflammation-related pathways such as NF-κB and STAT3. Finally, we validated an inflammatory microenvironment effect on GATA4 expression *in vivo* with nude mouse models of dibutyltin dichloride (DBTC)-induced pancreatitis and tumor xenografts.

## Materials and Methods

### PDAC Patient Samples

This study included PDAC patients that attended the Shanghai General Hospital, Shanghai Jiao Tong University School of Medicine for surgical resection. PDAC tumor tissue (*n* = 39) and non-cancerous tissues (*n* = 7) were frozen in liquid nitrogen and stored at −70°C for subsequent mRNA and protein analysis. The Research Ethics Committee of the Shanghai General Hospital, Shanghai Jiao Tong University School of Medicine, Shanghai, China approved this study, which followed the Helsinki Declaration. Informed written consent was provided by all patients.

### Cell Culture

The human PDAC cell lines, AsPC-1, BXPC-3, and PANC-1 (American Type Culture Collection, ATCC; Manassas, VA, United States), were cultured in Dulbecco’s modified Eagle’s medium (DMEM) containing 10% fetal bovine serum (FBS) and penicillin/streptomycin (100 units/mL) at 37°C in a humidified atmosphere of 5% CO_2_ and tested negative for the presence of mycoplasma. Human pancreatic duct epithelial (HPDE) cells (ATCC) were cultured in keratinocyte serum-free media with bovine pituitary extract and epidermal growth factor (Life Technologies, Waltham, MA, United States). THP-1 cells (ATCC) were stimulated with 0, 50, or 100 ng/ml of lipopolysaccharide (LPS) purchased from Enzo Life Sciences International (farmingdale, NY, United States) for 12 h. LPS-stimulated monocyte conditioned medium (LSMCM) was then used to activate PDAC lines for 0–96 h.

RETRACTED

### Immunohistochemistry

Sections (5 μm) of paraffin-embedded xenograft tissues were deparaffinized and rehydrated. They were then subjected to microwave antigen retrieval in EDTA antigen retrieval buffer, incubated with 3% hydrogen peroxide, and blocked with bovine serum albumin. Sections were incubated with primary antibodies against CD68 (1:8,000; Abcam, Cambridge, United Kingdom, ab213363), 163 (1:500; Abcam ab182422), GATA4 (1:1,600; Abcam ab84593), or Ki67 (1:200; Abcam ab16667). Staining was performed as described previously (Jimenez et al., 1999) and images were examined using Image ProPlus software (Media Cybernetics, Rockville, MD, United States).

### Cell Transfection

AsPC-1, BXPC-3, and PANC-1 PDAC cells were transfected with pEX-M35 empty vector and GATA4 expression vector (pEX-M35-GATA4) using Lipofectamine 2000 (Invitrogen, Carlsbad, CA, United States) following the manufacturer’s guidelines. The downregulation of GATA4 was achieved by using short hairpin RNA (shRNA) sequences (shGATA4-1#: 5′-TTCTCCGAACGTGTCACGT-3′; shGATA4-2#: 5′-GAATAAATCTAAGACACCA-3′; GenePharma, Shanghai, China). The scramble negative control shRNA was SCR: 5′-TTCTCCGAACGTGTCACGT-3′. Lentiviral production and transduction were performed by cloning sequences into the lentiviral pLKO.1 puro vector (GeneChem, Shanghai, China) following the manufacturer’s guidelines.

### Quantitative Reverse Transcription PCR (qRT-PCR)

Total RNA was prepared following a standard procedure using TRIzol reagent (Invitrogen). We synthesized cDNA from 1 μg RNA via MMLV reverse transcriptase (Invitrogen). The level of mRNA expression was determined with qRT-PCR using SYBR Green on a Bio-Rad CFX96 system (Hercules, CA, United States). Target gene expression was quantified using the cycle threshold (CT) method (2^–ΔΔ*ct*^) and each mRNA CT value was normalized to those of GAPDH. Experiments were performed in triplicate. The GATA4 primer sequences were 5′-CCTCTACCACAAGATGAACG-3′ (f) and 5′-CCTCTTTCCGCATTGCAAGA-3′ (r).

### Western Blot Analysis

Protein was extracted from PDAC cells using sample buffer (2% SDS, pH 6.8, 62.5 mmol/l Tris-HCl, 5% 2-β-mercaptoethanol, and 10% glycerol), cytosolic and nuclear extracts were prepared using NE-PER Nuclear and Cytoplasmic Extraction Reagents (Pierce Biotechnology) supplemented with a protease inhibitor cocktail kit (Pierce Biotechnology) according to the manufacturer’s instructions. Protein concentrations were determined using the BCA method (Thermo Fisher Scientific, Waltham, MA, United States). Total protein samples (30 μg) were separated on SDS polyacrylamide gels and transferred to polyvinylidene fluoride membranes (Millipore, Burlington, MA, United States). Membranes were incubated with primary antibodies against GATA4 (1:2,000, Abcam ab84593), GAPDH (1:500, Abcam ab8245), p-STAT3 (phospho Y705) (1:2,000, Abcam ab76315), STAT3 (1:1,000, Abcam ab68153), p65 (1:500, Abcam ab16502), p-p65 (phospho S529) (1:500, Abcam ab97726), β-actin (1:1000; Sigma-Aldrich, St. Louis, MO, United States, A2228), and histone H1(Proteintech Group). The anti-β-actin antibody was used as a loading control, Histone H1 indicates a nuclear protein internal control. Next, membranes were incubated with horseradish peroxidase-conjugated secondary antibodies. Immunoreactive protein bands were detected with enhanced chemiluminescence reagent (Thermo Fisher Scientific) and ImageJ software was used for quantification.

RETRACTED

### Cell Proliferation Assays

Cell proliferation was assessed with an MTT kit (Sigma-Aldrich) following the manufacturer’s instructions. Colony formation was assessed by seeding cells into six-well plates and culturing in media containing 10% FBS for 14 days. Emergent colonies were fixed with methanol, stained with 1% crystal violet (Sigma-Aldrich) and counted.

### Cell Migration and Invasion

PDAC cells (5 × 10^5^ per well) were seeded into 24-well Transwell plates coated with Matrigel (BD Biosciences, San Jose, CA, United States). cells were grown in the upper well of a Transwell chamber (8 μm pore size; Millipore, Burlington, MA, United States) and DMEM containing 10% FBS was added to the bottom chambers, cell were allowed to invade and migrate for 1 day. Cells were fixed and stained with crystal violet. Five random fields of cells that had passed into the lower surface were counted. The stained cells (migrating and invasive) were imaged and counted in five random fields for each sample. Each experiment was repeated three times independently.

### Immunofluorescence Microscopy

Cells were subjected to immunochemical staining through incubation with primary antibodies against GATA4 (1:50, Abcam ab194072) or CD68 (1:100, Abcam ab213363) overnight followed by incubation with AlexaFluor-conjugated secondary antibodies (1:1,000, Life Technologies). Nuclei were stained with DAPI. Fluorescence microscopy was used to observe cells.

### Animal Models

Animal experiments were performed in accordance with the Institutional Animal Ethics Committee Guidelines. To generate tumors, female BALB/c nude mice (aged 6 weeks) were injected subcutaneously with transfected cells, For orthotopic xenograft nude mouse model, we injected transfected cells into the body-tail of the pancreas of female BALB/c nude mice aged 6 weeks at a density of 1 × 10^6^ cells. After 1 week, DBTC (2 mg/kg) or DMSO (50 μl) was injected into the tail vein. Tumor size and volume were measured regularly. Mice were euthanized 6 weeks after implantation and tumors were resected for further analysis.

RETRACTED

### Statistical Analyses

All data are presented as mean ± SD. All experiments were repeated 3 times independently, Statistical analyses were conducted using GraphPad Prism software (La Jolla, CA, United States) and significance was denoted as *P* < 0.05. Statistical analysis between the two groups was analyzed by *t*-test and among more than two groups was conducted by one-way analysis of variance (ANOVA).

## Results

### GATA4 Is Related to Macrophages Infiltration in Pancreatic Cancer Tissues

The previous results showed that GATA4 expression was increased in PDAC (Karafin et al., 2009) and our results were consistent with it (Figures 1A–C), we examined GATA4 mRNA and protein expression levels in the tumor and adjacent tissue from PDAC patients. GATA4 mRNA levels were significantly higher in the tumor tissue compared to non-tumor controls (*P* = 0.0274), while GATA4 protein levels were also higher in the majority of paired tumor and non-tumor tissue samples (Figures 1A,B). These findings were validated by immunohistochemical staining (Figure 1C). In addition, Immunohistochemical staining analysis also showed significant enrichment of macrophages in the PDAC tissues compared to the adjacent normal pancreatic tissues (Figure 1C). Furthermore, hematoxylin and eosin (H&E) staining revealed the presence of pancreatic intraepithelial neoplasia (PanIN) in the tumor samples. PanIN lesions can be classified into three grades with respect to their morphology and degree of dysplasia, with the greatest dysplasia occurring in PanIN-3 (Hruban et al., 2001). Low-grade PanIN-1 and 2 lesions with nuclear crowding and variation in nuclear size were observed in DAPI-stained tissue (Figure 1D). Positive staining for CD68 indicated the presence of macrophages in the tumor environment. In addition, GATA4 was found to be highly expressed in the cytoplasm of tumor tissue, but was virtually undetectable in normal tissue.

**FIGURE 1:** GATA4 is upregulated in pancreatic cancer tissues. **(A,B)** GATA4 levels, detected by qRT-PCR and immunoblotting, were significantly upregulated in human PDAC patient samples (T: tumor tissues, N: adjacent non-tumor tissues). **(C)** Immunohistochemical staining for GATA4 and CD68 in PDAC tumors and matched normal adjacent tissue samples revealed increased levels of GATA4 and CD68 in PDAC tissue (original magnification, 200×). *P < 0.05. **(D)** Patient samples that contain PanIN1/2 lesions were stained with H&E (left panel), or were analyzed by immunofluorescence for GATA4 expression and the presence of macrophages (anti-CD68). DAPI stains nuclei. Scale bar, 50 μm.

RETRACTED

### Inflammatory Stimuli Promote the Invasion and Growth of Pancreatic Cancer Cells *in vitro*

To further investigate the effect of the immune system in pancreatic cancer invasion and growth, we examined the viability of three cancer cell lines (BXPC-3, AsPC-1, and PANC-1) stimulated with lipopolysaccharide (LPS)-stimulated monocyte conditioned medium (LSMCM) for up to 96 h. LSMCM was obtained from the human monocyte cell line THP1 (Tsuchiya et al., 1980) stimulated with LPS (0, 50, and 100 ng/ml) for 12 h. Cells treated with LSMCM had a significantly higher dose-dependent viability after 96 h than untreated cells (*P* < 0.01; Figure 2A). Similarly, significantly increased colony formation was observed in the three cell lines following 1 day of treatment with LSMCM (Figure 2B). The Transwell assay was used to examine the migration and cell invasion properties of the three cell lines after 1 day exposure to LSMCM. We found a dose-dependent increase in cell invasion and migration, which was significant at the highest concentration of LPS treatment (*P* < 0.05; Figure 2C). Taken together, our findings suggest that inflammatory stimuli promote pancreatic cancer invasion and growth *in vitro*.

**FIGURE 2:** Inflammatory stimuli promote the growth and invasion of pancreatic cancer cells *in vitro*. **(A)** MTT assay measuring cell viability of three pancreatic cancer cell lines (BXPC-3, PANC-1, and AsPC-1) incubated with lipopolysaccharide (LPS) stimulated monocyte conditioned medium (LSMCM) for 24, 48, 72, and 96 h. LSMCM was obtained from THP1 cells stimulated with LPS (0, 50, and 100 ng/ml) for 12 h. **(B)** Colony formation is increased in a dose-dependent manner in cells following LSMCM treatment for 24 h. Colony formation was determined by crystal violet staining and quantified by counting the number of colonies after 2 weeks. **(C)** The Transwell assay was used to examine cell migration and invasion following 24 h exposure to LSMCM. Cells that had migrated to the lower membranes were photographed and quantified under 400× magnification. The data are presented as the mean ± SEM. *P < 0.05 and **P < 0.01.

### Inflammatory Stimuli Promote GATA4 Expression in Pancreatic Cancer Cell Lines

Previous studies have pointed out the expression of GATA4 in PDAC cell lines (Karafin et al., 2009). In this experiment, GATA4 expression levels in three PDAC cell lines (BXPC-3, AsPC-1, and PANC-1) were examined by qRT-PCR and western blot analyses, and compared to normal pancreatic HPDE cells. PANC-1 and AsPC-1 cells had significantly higher levels of GATA4 mRNA expression than normal pancreatic HPDE cells (both *P* < 0.01). BXPC-3 cells had lower GATA4 mRNA expression than PANC-1 and AsPC-1 cells (Figure 3A), but higher GATA4 protein expression (*P* < 0.01; Figure 3B), which was consistent with the results of previous studies (Karafin et al., 2009). Furthermore, although GATA4 protein levels were lower in AsPC-1 and PANC-1 cells than BXPC-3 cells, they were still significantly higher than in normal pancreatic cells. GATA4 mRNA and protein levels were also analyzed in three cell lines incubated with LSMCM obtained by treating THP1 cells with increasing concentrations of LPS (Figures 3C–H). GATA4 mRNA expression increased dose-dependently in response to inflammatory stimuli in all three cell lines. Similarly, GATA4 protein levels were significantly higher in all three cell lines, with the highest increase observed in response to treatment with the highest dose of LPS (*P* < 0.01). These results indicate that GATA4 has a similar profile *in vitro* to that observed in human PDAC tissue.

RETRACTED

**FIGURE 3:** GATA4 expression is increased in pancreatic cancer cell lines. **(A,B)** GATA4 mRNA and protein levels were measured by qRT-PCR and western blotting, respectively and found to be higher in the pancreatic cancer cell lines (BXPC-3, PANC-1, and AsPC-1) compared to a normal pancreatic cell line HPDE. GAPDH was used as a loading control. GATA4 mRNA and protein expression levels were also detected by qRT-PCR and immunoblotting, respectively, in BXPC-3 **(C,D)**, PANC-1 **(E,F)**, and AsPC-1 **(G,H)** incubated with LSMCM for 24 h. The data are presented as mean ± SEM. *P < 0.05 and **P < 0.01.

### Effects of GATA4 Knockdown on Proliferation, Colony Formation, Invasion, and Migration of Cell Exposed to LSMCM *in vitro*

We next sought to determine whether GATA4 suppression could affect migration, proliferation and invasion of pancreatic cancer cell exposed to LSMCM. PANC-1 and BXPC-3 cell lines were stably transfected with either shGATA4-1/2 or a scrambled vector. qRT-PCR were used to examine the transfection efficiency of GATA4 (Figures 4A,B), Cell viability was decreased in both PANC-1 and BXPC-3 cells when GATA4 expression was suppressed (Figures 4C,D). And GATA4 expression was increased following incubation with LSMCM (Figures 4E,F), Moreover, the colony-forming ability of PANC-1 and BXPC-3 GATA4-knockdown cells was decreased following incubation with LSMCM (Figures 4G,H), although the number of colonies was significantly increased in the scrambled control shRNA-treated cells. Thus, GATA4 knockdown inhibits colony formation and cell proliferation in pancreatic cancer cells *in vitro*. However, studies have pointed out that reduction of GATA4 significantly increased the colony formation ability of both of pancreatic cancer cell lines (Gong et al., 2018), cell exposed to LSMCM may have caused this difference. Similar results were obtained in the invasion and migration assays. GATA4 suppression in either PANC-1 or BXPC-3 cells exposed to LSMCM reduced cell migration and invasion, while significantly increased migration and invasion was observed in the scrambled control shRNA-treated cells (Figures 5A–D).

RETRACTED

**FIGURE 4:** GATA4 knockdown inhibits cell proliferation and colony formation *in vitro*. **(A,B)** The expression of GATA4 in different treatments by qRT-PCR, *P < 0.05 and **P < 0.01. **(C,D)** Pancreatic cancer cells BXPC-3 and PANC-1 were stably transfected with shGATA4-1/2 or scramble shRNA as indicated for 48 h. Cell viability was tested in GATA4-shRNA expressing cells using an MTT assay at 24, 48, 72, and 96 h. **(E,F)** The expression of GATA4 in different treatments by western blot. **(G,H)** Colony formation was decreased in GATA4 knockdown cells following incubation with LSMCM for 24 h. Colony formation was determined by crystal violet staining and quantified by counting the number of colonies 2 weeks later.

**FIGURE 5:** GATA4 knockdown inhibits cell migration and invasion *in vitro*. BXPC-3 **(A,B)** and PANC-1 **(C,D)** cells were exposed to LSMCM for 24 h. Cell migration and invasion were determined by a Transwell assay using crystal violet staining. Cells that had migrated to the lower membranes were photographed and quantified under 400× magnification. The data are presented as the mean ± SEM. *P < 0.05 and **P < 0.01.

### GATA4 Overexpression Promotes Invasion and Migration of Cells Following Incubation With LSMCM Stimulated by Varying Concentrations of LPS *in vitro*

To examine the effects of GATA4 overexpression on migration, proliferation, colony formation and invasion of cells following incubation with LSMCM stimulated by varying concentrations of LPS, GATA4 was ectopically expressed in AsPC-1 cells. Cell viability and colony-formation were significantly increased in GATA4-overexpressing cells following incubation with LSMCM stimulated by varying concentrations of LPS (Figures 6A,C). However, previous studies showed that GATA4 over-expression reduced cell proliferation and colony formation in pancreatic cancer cells (Gong et al., 2018). The reason for the difference between our results and Gong et al. may be that pancreatic cancer cells were treated with LSMCM. The specific reasons need to be further studied. Western blot results showed that GATA4 expression increased after LPS stimulation (Figure 6B). Likewise, cell migration and invasion were increased by GATA4 overexpression (Figures 6D,E). Overall, our findings demonstrate that GATA4 knockdown suppressed migration, proliferation, colony formation and invasion of cells following incubation with LSMCM *in vitro* while overexpression promoted these characteristics.

RETRACTED

**FIGURE 6:** GATA4 overexpression promotes cell proliferation, colony formation, migration, and invasion. **(A)** GATA4 was ectopically expressed in AsPC-1 cells. Cell viability was detected using an MTT assay at 24, 48, 72, and 96 h. **(B)** The expression of GATA4 in different treatments by western blot. **(C)** Colony formation was increased in GATA4 overexpressing cells following incubation with LSMCM for 24 h. Colony formation was determined by crystal violet staining and quantified by counting the number of colonies after 2 weeks. **(D,E)** Cell migration and invasion were determined by a Transwell assay using crystal violet staining. GATA4 overexpression aggravates cell migration and invasion. Cells that had migrated to the lower membranes were photographed and quantified under ×400 magnification. The data are presented as the mean ± SEM.*P < 0.05 and **P < 0.01.

### GATA4 Exacerbates Inflammation-Driven PDAC Progression via NF-κB and STAT3 Signaling Pathways

To elucidate the signaling pathways that may be affected by the differential expression of GATA4, we analyzed levels of nuclear and total p65, a NF-κB activation marker (Maguire et al., 2011). Since the JAK-STAT3 signaling pathway is thought to promote tumorigenesis through inflammation (Yu et al., 2014), First, the purity of the obtained fractions was verified by western blotting (Figure 7A), then we examined the phosphorylation status of STAT3. We found that suppression of GATA4 in PANC-1 and BXPC-3 cells resulted in decreased levels of nuclear p65 and phosphorylation of STAT3 (Figures 7B,C). However, LSMCM treatment reversed this trend to some extent. Furthermore, overexpression of GATA4 in AsPC-1 cells led to an increase in nuclear p65 levels and phosphorylation of STAT3, especially when cells were treated with LSMCM (Figure 7D). These findings indicate that GATA4 may participate in the PDAC inflammation-driven progression via the NF-κB and STAT3 signaling pathways.

**FIGURE 7:** GATA4 exacerbates inflammation-driven PDAC progression via NF-κB and STAT3 signaling pathways. Three cell lines were cultured with LSMCM for 24 h. **(A)** Western blots was used to verify the purity of fractions obtained from the cell fractionation. lactate dehydrogenase indicates cytosol. Histone H1 indicates nuclei. **(B–D)** Western blot analysis was performed to determine the expression and phosphorylation of the indicated proteins, Histone 1 indicates a nuclear protein internal control.

RETRACTED

### Differential Expression of GATA4 in Pancreatic Cancer Cell Growth Stimulated by DBTC *in vivo*

Differential expression of GATA4 was assessed in nude mice subcutaneously injected with PANC-1 cells with or without stable shGATA4 expression. After 1 week, chronic pancreatitis was induced by DBTC and the size of xenograft tumors was monitored for 28 days. Suppression of GATA4 resulted in reduced xenograft tumor growth (Figure 8A). The inflammation induction effect of DBTC was first confirmed (Figure 8B). H&E staining of pancreatic orthotopic xenografts confirmed that chronic pancreatitis had been induced by DBTC and that cells were irregular with varying nuclear sizes. However, these characteristics were less pronounced when GATA4 was suppressed, Using immunohistochemistry and the macrophage marker CD68, we proved that treatment of DBTC induced macrophage infiltration, indicating the successful establishment of the chronic pancreatitis model by DBTC injection (Figure 8B). Immunohistochemistry indicated that CD68, CD163, Ki67, and GATA4 levels were increased after DBTC but GATA4 knockdown reduced these effects (Figure 8B). Next, we continued to explore the influence of GATA4, on metastasis *in vivo*, The results showed that GATA4 knockdown reduced liver metastases (Figure 8C). Western blotting indicated that the levels of nuclear p65 and phosphorylated STAT3 were reduced when GATA4 expression was inhibited (Figure 8D). However, DBTC-induced pancreatitis led to an increase in nuclear p65 and phosphorylated STAT3 protein expression (Figure 8D). These data indicate that GATA4 knockdown attenuates pancreatic cancer cell growth stimulated by inflammatory factors *in vivo*.

**FIGURE 8:** | Knockdown of GATA4 attenuates pancreatic cancer cell growth stimulated by inflammation *in vivo.* **(A)** Tumor growth was assessed in nude mice that were subcutaneously injected into the right axilla with 1 × 10^6^ PANC-1 cells with or without stable shGATA4 expression. After 1 week, dibutyltin dichloride (DBTC, 2 mg/kg) or DMSO was injected into the mice tail vein of each subgroup (*n* = 6 per group). Subsequently, the xenograft tumor size was monitored every week (volume = width^2^ × length × 1/2). Points represent the mean tumor volumes of three independent experiments. After 28 days, the xenograft tumors were excised from the mice. **(B)** Pathological and immunohistochemical examination of pancreatic orthotopic xenografts. Immunohistochemistry was performed using antibodies targeting CD68, CD163, Ki67, and GATA4. Arrows indicate macrophages. Scale bar, 50 μm. **(C)** Macroscopic photos of mouse liver tissues (upper panel) and HE staining of metastatic nodules in livers (lower panel). **(D)** The expression and phosphorylation status of the NF-κB and STAT3 signaling pathway proteins were detected in the xenograft tumors by immunoblotting assays. The data are presented as mean ± SEM. *P < 0.05 and **P < 0.01.

RETRACTED

In contrast to the reduction of tumor growth observed when GATA4 expression is suppressed, overexpression of GATA4 promoted tumor growth in our mouse model of chronic pancreatitis (Figure 9A). Immunohistochemical and pathological examination of pancreatic orthotopic xenografts found that levels of CD68, CD163, Ki67, and GATA4 were elevated when GATA4 was overexpressed (Figure 9B). The expression and phosphorylation status of STAT3 as well as the NF-κB signaling pathway were the highest in xenograft tumors overexpressing GATA4 (Figure 9C). Overall, these results demonstrate that GATA4 exacerbates pancreatic cancer cell growth stimulated by pancreatic inflammation *in vivo*.

**FIGURE 9:** GATA4 exacerbates pancreatic cancer cell growth stimulated by inflammation *in vivo.* **(A)** Tumor growth was assessed in nude mice that were subcutaneously injected into the right axilla with 1 × 10^6^ AsPC-1 cells with or without stable GATA4 expression. After 1 week, dibutyltin dichloride (DBTC, 2 mg/kg) or DMSO was injected into the mice tail vein of each subgroup (*n* = 6 per group). Subsequently, the xenograft tumor size was monitored every week (volume = width^2^ × length × 1/2). Points represent the mean tumor volumes of three independent experiments. After 28 days, the xenograft tumors were excised from the nude mice. **(B)** Pathological and immunohistochemical examination of pancreatic orthotopic xenografts. Immunohistochemistry was performed using antibodies against CD68, CD163, Ki67, and GATA4. Arrows indicate macrophages. Scale bar, 50 μm. **(C)** The expression and phosphorylation status of the NF-κB and STAT3 signaling pathway proteins were detected in the xenograft tumors by immunoblotting assays. The data are presented as mean ± SEM. *P < 0.05 and **P < 0.01.

## Discussion

The association between PDAC and inflammation has led to the development of novel therapeutics that target inflammatory factors (Steele et al., 2016; Shadhu and Xi, 2019). However, since many of these therapeutics are limited by multiple off-target effects and lack of specificity (Zhu et al., 2018), the development of more appropriate therapies is an ongoing process. In the present study, we confirm that GATA4 expression influences cancer progression via the inflammation-related pathways NF-κB and STAT3.

RETRACTED

We found that GATA4 was overexpressed in PDAC tissue as well as in three PDAC cell lines (PANC-1, AsPC-1, and BXPC-3). GATA4 expression levels varied between the three cell lines with the highest mRNA levels observed in PANC-1 cells followed by the AsPC-1 cell line. Although GATA4 mRNA levels were lower in BXPC-3 cells, GATA4 protein levels were significantly higher in BXPC-3 cells, perhaps indicating that the protein was not degraded in these cells. GATA4 is known to accumulate in multiple tissues as a consequence of aging and associated inflammation (Kang et al., 2015). PANC-1 cells are derived from the PDAC primary tumor of a 56 year old female (Lieber et al., 1975), AsPC-1 from the ascites of a 62 year old female (Chen et al., 1982), and BXPC-3 from the primary tumor of a 61 year old female (Tan et al., 1986). Interestingly, BXPC-3 cells have been shown to have significantly higher cyclooxygenase-2 (COX2) levels than the other two cell lines (Deer et al., 2010). COX2, a prostaglandin that activates factors involved in angiogenesis (Masferrer et al., 2000), is known to be upregulated by NF-κB (Poligone and Baldwin, 2001). NF-κB is thought to be regulated by GATA4 to initiate a senescence-associated secretory phenotype, which is described as a proinflammatory response linked to the promotion of tumorigenesis and aging (Kang et al., 2015). Senescence-associated inflammation induced by KRAS and the histone deacetylase-associated protein SIN3B has been found to positively correlate with PDAC progression (Rielland et al., 2014). GATA4 is known to promote the expression and secretion of proinflammatory cytokines in senescent cells, which can then stimulate neighboring malignant cells into proliferation to form tumors (Krtolica et al., 2001). Therefore, the high expression of GATA4 in BXPC-3 cells could be the consequence of a phenotype that promotes the release of proinflammatory cytokines and tumorigenesis, which perhaps activates KRAS-induced senescence. Our results emphasize the heterogeneity in PDAC and highlight the difficulties in identifying pathways that behave similarly in every cell line. Certainly, the interactions involving GATA4 and NF-κB in BXPC-3 cells warrant further investigation.

In the current study, the extent of STAT3 and NF-κB signaling in the differential expression of GATA4 was analyzed by measuring levels of nuclear p65, a marker of NF-κB activation, and the phosphorylation status of STAT3. We found that suppression of GATA4 results in a reduction of nuclear p65 levels and STAT3 phosphorylation. However, the presence of LPS-induced inflammatory stimuli reversed this trend. Furthermore, overexpression of GATA4 enhanced the activation of NF-κB and STAT3. These findings suggest that GATA4 may participate in the NF-κB and STAT3 signaling pathway in response to inflammatory mediators. Moreover, we found that inflammatory stimuli and the differential expression of GATA4 can influence migration and cell invasion. Several studies have observed similar results with STAT3 and NF-κB signaling in relation to inflammation and the transition from chronic pancreatitis to PDAC (Baumgart et al., 2014; Loncle et al., 2015; Tao et al., 2016). Loncle et al. (2015) demonstrated that the JAK2–STAT3-dependent pathway was activated by IL-17 and REG3β, a mediator of pancreatitis and PanIN lesions, to promote cell growth. Inactivation of REG3b in KRAS-driven PDAC was shown to reduce the formation of PanIN. Moreover, the downregulation of NF-κB and STAT3 signaling has recently been reported to increase pancreatic cancer cell sensitivity to chemotherapy (Gong et al., 2017). The combined targeting of STAT3/COX-2/NFκB/EP4 could effectively manage the progression of pancreatic cancer, as reduced levels of STAT3 and NFκB resulted in the transcriptional suppression of COX-2 and reduced the level of fibrosis induced by the prostaglandin receptor EP4 (Gong et al., 2014). However, inhibition of either STAT3 or NFκB alone did not effectively control tumor progression. The inhibition of STAT3 led to elevated levels of NFκB indicating that STAT3 inhibitors alone may not effectively control disease progression (Gong et al., 2014). Nevertheless, several STAT3 inhibitors are currently being developed with some reaching early stage clinical trials (Oh et al., 2015; Bai et al., 2018; Reilley et al., 2018). Certainly, the interactions between GATA4, STAT3, NFκB, KRAS, and COX2 should be investigated further through co-immunoprecipitation studies in the three different cancer cells (PANC-1, AsPC-1, and BXPC-3) in the absence or presence of LSMCM.

RETRACTED

## Conclusion

In conclusion, our results validate the involvement of inflammation in PDAC progression and indicate that GATA4 overexpression aggravates inflammatory stimuli-induced pancreatic cancer cell invasion and growth via NF-κB and STAT3 signaling pathways. Overall, we present a mechanism of inflammation-driven cancer progression that is dependent on GATA4 expression via NF-κB and STAT3 signaling, which may lead to the development of novel therapeutic interventions.

## Data Availability Statement

The raw data supporting the conclusions of this article will be made available by the authors, without undue reservation.

## Ethics Statement

The Research Ethics Committee of the Shanghai General Hospital, Shanghai Jiao Tong University School of Medicine, Shanghai, China approved this study. The patients/participants provided their written informed consent to participate in this study. We performed animal experiments following the Institutional Animal Ethics Committee Guidelines.

## Author Contributions

WJ, CC, and LH performed the experiments, acquired the data, and drafted the manuscript. LY revised the manuscript critically for important intellectual content and substantially contributed to the conception and design of this study. JS analyzed and interpreted data. All authors read and approved the final manuscript and agreed to be accountable for all aspects of the research in ensuring that the accuracy or integrity of any part of the work are appropriately investigated and resolved.

## Conflict of Interest

The authors declare that the research was conducted in the absence of any commercial or financial relationships that could be construed as a potential conflict of interest.
